The article "Art-Based Workshops for Women: An Opportunity for Reflection on Identity and Transformation following Cancer Treatment" was published in 2023. Journal: Occup Ther Int.

# Art-Based Workshops for Women: An Opportunity for Reflection on Identity and Transformation following Cancer Treatment

**DOI:** 10.1155/2023/1828314

**Published:** 2023-07-17

**Authors:** Marie-Christine Ranger, Sandra Houle, Alysson Rheault, Roanne Thomas

**Affiliations:** School of Rehabilitation Sciences, University of Ottawa, Ottawa, Canada K1H 8L1

## Abstract

Individuals experiencing cancer often report feelings of abandonment by the healthcare system after medical treatment has ended. Specifically, women with cancer have expressed the need for support beyond traditional medical and rehabilitation periods, especially with the process of reconstructing the self in the context of enduring illness. Occupational therapists could play a critical role in providing opportunities for self-reflection and transformation through occupation for this population. Art-based occupations may be especially useful for providing space for self-reflection and personal change. This article describes the experiences of women living with cancer who participated in community art-based workshops that focused on the themes of identity and transformation. The project consisted of mixed-media workshops that were held at a community-based facility providing supportive programs for people living with cancer. Eleven women participated in the workshops led by an art-based rehabilitation researcher and a visual artist. Workshops were audio-recorded, and photographs of the participants' artwork were taken. Individual postworkshop interviews were conducted with the participants, within 4 to 6 weeks following the last workshop. Interpretive description was used to capture four themes with implications for personal change, transformation, and occupational therapy: (1) revealing: therapeutic potential; (2) sharing: vulnerability and new perspectives; (3) transforming: the self; and (4) creating: regular practices. The findings point to ways occupational therapists can form new partnerships with other disciplines and professionals to generate positive outcomes for people living with cancer.

## 1. Introduction

The lifetime probability of developing some form of cancer for Canadian women is estimated at 1 in 2.4 or 43% [1]. Due to significant efforts in cancer prevention and screening, as well as investments in detection and treatment, mortality rates have been declining steadily in Canada [2]. From a medical perspective, completing cancer treatments is generally thought of as the final chapter in the cancer experience; yet, the consequences of living with and beyond cancer are complex, and often enduring [3]. Individuals frequently face hardships related to dealing with acute and long-lasting symptoms, navigating a complicated healthcare system, and reconciling with changing identities and roles [4]. A lack of support in the process of understanding and adapting to one's personal experience of living with an illness [5], especially beyond acute cancer treatment, can lead to unnecessary suffering and feelings of abandonment by the healthcare team [3, 6, 7].

The article "Art-Based Workshops for Women: An Opportunity for Reflection on Identity and Transformation following Cancer Treatment" was published in 2023. Journal: Occup Ther Int.

Occupational therapists (OT) have a unique set of skills and a body of knowledge to support the range of issues faced by individuals living with and beyond cancer [8]. Yet, the role of occupational therapists with these individuals remains generally underresearched [7, 9] and underutilized [3, 8]. Recently, certain occupational therapy scholars have focused on the potential for clinicians to foster positive experiences of personal change and transformation through occupation with individuals living with long-term health conditions [10]. Specifically, art-based occupations have been shown to foster reflection and reimagining of the self in participants who experience cancer [6, 11, 12], which are key aspects of a positive transformative process [13].

Biographical disruption occurs when one's sense of self and identity is threatened by illness or disability [14]. Experiences of biographical disruption in individuals living with and beyond cancer may stem from a disruption to daily life that continues past treatment, the untiring threat of reoccurrence, a heightened sense of one's own mortality, and a loss of one's anticipated life course [15]. Specifically, women describe a sense of vulnerability following the end of treatment where a process of reinventing themselves and accepting their new normal is critical [16]. Furthermore, women may experience disruption related to very specific gender-determined identities and roles. For example, in a metasynthesis of the impact of undergoing a mastectomy, Sun et al. found that participants experienced a feeling of a discrepancy between their self-image and the expected societal image of a woman, leading to experiences of stigma, psychological distress, and social isolation [17]. The individualized experiences of these women were expressed against their collective need to address, cope, and adapt to their new sense of self [17]. Importantly, however, the findings of this study also describe the experiences of some women who saw their mastectomies as a chance to start over, discard the body part that no longer served them, and resist societal demands of women's bodies. Thus, the experience of biographical disruption due to living with or beyond cancer may, for some, lead to positive personal changes, adaption, and transformation of the self [15].

The article "Art-Based Workshops for Women: An Opportunity for Reflection on Identity and Transformation following Cancer Treatment" was published in 2023. Journal: Occup Ther Int.

Evidently, women living with cancer often experience an ongoing need to reflect on their illness experiences and identity to reconcile disruptions caused by the experience of cancer. However, they are rarely provided with the opportunity and support to do so in current health care and rehabilitation care settings [18]. When occupational therapists are involved in the care of this population, they are generally referred to address acute cancer issues. For example, occupational therapists typically provide educational programs, inform clients about relaxation techniques and management of fatigue, or work toward enhancing specific skills, such as hand, upper limb, or cognitive function [9].

Dubouloz Wilner studied extensively how occupational therapists can support clients in their need to reflect and reimagine the self through occupation [13, 19]. Adapting the theory of transformative learning to physical rehabilitation, Dubouloz Wilner describes how individuals living with various chronic illnesses, including cardiac issues, rheumatoid arthritis, and multiple sclerosis, undergo a process of deconstructing and reconstructing the self; allowing them to cope, manage, and adapt to these life-altering illnesses; and potentially leading to the development of a more authentic self [13, 19]. She refers to meaning perspectives in the context of transformation to include beliefs, values, feelings about one's identity, and experience of illness. Transformation occurs when new meaning perspectives are developed or previously held meaning perspectives are adjusted or completely reconstructed, enabling changes in a person's worldview. From this perspective, transformation is both a process and an outcome. Given that occupations are at once a reflection of our identity and a means for self-expression [20, 21], individuals who have lived through a severe illness reconstruct their daily lives by redefining values and meanings in their occupations [22]. Certain occupations can be especially useful to support a positive transformation in the experience of illness [19].

Art-based occupations can be a catalyst for self-reflection and exploration for individuals living with or beyond cancer, which can lead to positive personal change and transformation [11, 23]. In a qualitative study, Reynolds and Prior described how women living with cancer experienced a state of “deep immersion” or flow while participating in creative occupations which facilitated a sense of control and psychological growth [11]. Flow is a well-established concept in occupational therapy, where it is defined as the psychological state of being completely absorbed in a rewarding occupation, to the point of losing the sense of time [24]. According to Hansen et al., art-based occupations consist of elements of art and craft that require the use of mind and body and are experienced as meaningful [25]. Working with multiple art materials allows individuals to explore a wide range of experiences and feelings [23]. Furthermore, art-based occupations can facilitate self-expression when such emotions are complex and challenging to put into words [26, 27]. By offering various possibilities to reflect on identity and explore different avenues for self-expression, occupational therapists can provide opportunities for clients to reimagine a new self [25, 26]. Furthermore, having the opportunity to choose how best to express oneself can be experienced as an opportunity to regain personal control over one's occupations, which may have been diminished previously through the illness experience [26, 28]. Finally, when used in a group setting, art-based occupations can facilitate exchanges by focusing the discussion on the creative process [28, 29] which is perceived as less threatening than a discussion-based peer support group [23].

The article "Art-Based Workshops for Women: An Opportunity for Reflection on Identity and Transformation following Cancer Treatment" was published in 2023. Journal: Occup Ther Int.

Despite their potential, a lack of research remains regarding the use of art-based occupations in occupational therapy and specifically with individuals living with or beyond cancer [11, 23, 30]. Therefore, the objective of the study was to describe the experiences of women living with cancer in community art-based workshops, with a focus on identity and transformation.

## 2. Positionality Statement

The two first authors are occupational therapists (OT) who have worked with various populations in the Canadian provinces of Quebec and Ontario and who have always been curious about the potential of art-based methods and creative occupations in practice. As doctoral students in the rehabilitation sciences program, we were exposed to and involved in the principal investigator's research on art-based community workshops for women with cancer. We believed that it was valuable to analyze the data from an OT perspective given its occupation-centred intervention. This article is a secondary analysis from an OT lens, of a study reported elsewhere [31]. Both occupational therapists were involved in the data analysis.

## 3. Materials and Methods

With the aim of enhancing the well-being of women living with cancer, two series of art-based community workshops were offered in a Regional Cancer Foundation Centre in Ottawa, Canada, to 11 women who live with cancer. Mixed-media art-based activities were proposed.

This study was approved by the University of Ottawa's Research Ethics Board. All participants provided their consent for their involvement in the study. Research participants were recruited via local cancer networks, using a method of snowball sampling. Women were eligible if they were 18 years of age or older, had completed active treatment for cancer or were well enough to attend, were comfortable speaking and writing in English, and were able to consent.

The article "Art-Based Workshops for Women: An Opportunity for Reflection on Identity and Transformation following Cancer Treatment" was published in 2023. Journal: Occup Ther Int.

### 3.1. Participants

The study consisted of two series of three mixed-media workshops (six workshops in total) led by an art-based rehabilitation researcher (the principal investigator) and a visual artist. A total of 11 women participated. Six women participated in the first workshop series. Of these participants, five returned for the second workshop series. An additional five women were recruited for a total of 10 participants in the second series. All materials were provided to participants, and no costs were incurred.  Table 1 presents a description of the participants.

### 3.2. Mixed-Media Art Workshops

Workshops were held at a community-based facility providing supportive programs for people living with cancer at all stages of illness. Workshops lasted from 3 to 4 hours. Each series was delivered over 3 weeks.

Mixed-media art involves a combination of techniques and materials, for example, building texture, layering paint, images, photo transfers, and other dynamic combinations. See Figures 1 and 2 for examples of mixed-media projects by workshop participants. The theme for the first workshop series was *Wabi sabi*, which is commonly defined as finding beauty in imperfection and transience. The participants' feedback from the first workshop was overwhelmingly positive. Therefore, a similar format was used during the second workshop series. For the second workshop series, the theme was *texturing small changes*. It was an exploration of the use of multiple layers. Both themes were chosen to alleviate participant concerns about creating “perfect” art.  Table 2 offers a description of each workshop series.

### 3.3. Data Analysis

During the final workshops of the series, photographs of participants' artwork were taken with the participants' consent. Individual interviews were conducted by telephone with each participant within 4 to 6 weeks after the last workshop.  Table 3 contains sample postworkshop interview questions. All workshops and interviews were audio-recorded and transcribed verbatim. These files were reviewed for accuracy by a research assistant. The text and photographs of the participants' artwork were interpreted together as the analysis proceeded. The transcripts were read holistically and line by line to extract significant statements following established guidelines for interpretive description [32]. To ensure the rigour of our analysis, we used a combination of qualitative digital analysis program (NVivo) and nondigital coding (i.e., on paper) [33]. First, three researchers independently coded the same transcripts and then different transcripts, to establish an initial coding structure based on shared discussions of our analyses before continuing to code in NVivo. Selected themes discussed herein were then reviewed further before writing.

The article "Art-Based Workshops for Women: An Opportunity for Reflection on Identity and Transformation following Cancer Treatment" was published in 2023. Journal: Occup Ther Int.

### 3.4. Processes

Table 4 illustrates the processes by which the facilitators acknowledged the individuality of each participant and encouraged their reflection and introspection. The facilitators' quotations offer glimpses into the workshop environment. It was intended to be a safe space, where participants were encouraged to explore, create, learn, and share. This provides the context for understanding the participant data presented in the findings section of the article.

## 4. Findings

Four interconnected themes emerged from the data. These themes illustrate aspects of cancer survivorship and personal change, as well as understandings of the self and meaningful occupation. They are the following: (1) revealing: therapeutic potential; (2) sharing: vulnerability and new perspectives; (3) transforming: the self; and (4) creating: regular practices.

### 4.1. Theme 1—Revealing: Therapeutic Potential

During the postworkshop interviews, all participants indicated that they found the art-based activities proposed during the workshop to be appealing (we use the term “arts-based activities” when referring to the activities provided during the workshops as a general descriptive category as opposed to the term “arts-based occupations” which are given a specific meaning by an individual). The level of engagement in the activities is apparent in participants' discussions of exploration and discovery, as well as their reflections on the ways in which time moved quickly during the workshops .

With respect to discovery, some participants were aware that they were exploring and expressing aspects of the self, while others were caught by surprise. The following participant eloquently explained how working with creative material allowed for an exploratory process which eventually led to the expression of something essential about the inner self:

When we do things intuitively, we discover things. Things percolate up through the art and we can reflect on it and it enriches us. (…) Because that's the idea, to have personal stuff come up and that's the revelation, that's what keeps you doing more of this stuff. But not just playing with colours and things and creating but what… what it reveals about you. (Patricia, S2I) (With respect to the interview data, pseudonyms are followed by the number of the workshop series (S1 or S2) and “I” indicates the data were from an interview. As is common in qualitative research wherein groups are recorded, individual participants are not identified. However, the workshop series (S1, S2) and the workshop number (W1, W2, W3) are noted.)

The article "Art-Based Workshops for Women: An Opportunity for Reflection on Identity and Transformation following Cancer Treatment" was published in 2023. Journal: Occup Ther Int.

For her part, Lynn shared how she surprised herself by getting completely involved in the art-based activity, to the point that she lost track of time. Lynn identified her state of flow as being caused by the infinite decisions she was making regarding how to express her true self through her artwork. Participants had access to an abundance of materials, colours, and textures with which to work. She related her creation to herself; the use of the word “unique” describes both the experience and her individuality:

The facilitator said, “Okay, we're going to start, and we have two hours,” and at one point I thought, “Boy, is it really going to take that long to do this?” But by the time I kept looking at the clock, I thought, “Wait a minute, I might run out of time here.” So it was really amazing, but I think it was because I was making so many little decisions and thoughtfulness about what I wanted this piece to be and it was an expression of me. I mean, that was really unique. Very unique. (Lynn, S1I).

In the first workshop of the second series, a participant reflected on the benefits of using art-based activities, which revealed the therapeutic potential of such activities. She emphasized how it is through the act of creating that the self is expressed and can subsequently be attended to. The art-based activity appeared to allow expression beyond words. The participant explained “Sometimes what gets expressed is stuff that I can't put into words. And it's only in doing that comes up with how I feel.” (S2, W1).

In her postworkshop interview, Erin also described the workshops as potentially therapeutic. Participants were invited to stitch a cotton bag to hold photos and small mementos. In the second step of the process, all the participants' bags were submerged in a turmeric dye bath. Finally, the bags were opened to reveal their altered content.  Figure 3 represents the content of a stitched cotton bag after the turmeric bath. In the participant's description of the outcome, one can imagine how the altered cloth and contents could be a stand-in for herself. She also hints at trusting the transformation that took place because it yields unexpected positive results:

I think that even the bag, the physical change of the bag after we soaked it. It was kind of powerful, you know, just to see that things change, they come out, they are different, but they are still really cool and still really beautiful. (Erin, S2I).

The article "Art-Based Workshops for Women: An Opportunity for Reflection on Identity and Transformation following Cancer Treatment" was published in 2023. Journal: Occup Ther Int.

Thus, the potential therapeutic aspects of the workshops were revealed through flow, as well as discussions of experiences that are not easily expressed in words and via the acceptance of change through altered objects.

### 4.2. Theme 2—Sharing: Vulnerability and New Perspectives

Participants indicated that creating alongside women with similar experiences with cancer added a reassuring element to the workshops. With care not to impose discussion, both facilitators encouraged the women to share their ideas regarding their artwork at the end of each workshop. Patricia stated how she found the words to share her thoughts and feelings with participants made her vulnerable but at the same time heightened the experience of the workshops. The commonality of the cancer experience was reassuring:

Some parts I really liked [for example] when we debriefed and showed each other our [artwork]. I thought that was really valuable. I found a lot of stuff came out of that and it was very moving and people were quite open actually in expressing themselves. I think that's a nice exercise because it reminds us the importance of doing that and being vulnerable. And kind of naming whatever is going on with us, whatever we have expressed through the art. It's nice to put words to it and, you know, because we have expressed it visually and by putting words to it, it's not always easy but to have that option it kind of closes the deal. (Patricia, W2I).

Participants were faced with multiple choices and decisions in the art-making process, which allowed them to move out of their comfort zone. As Lynn suggested, the challenge of experimenting with different materials benefited her creative work. She implies that the same lesson can relate to her everyday life and possibly to her experience of living with cancer—a new perspective:

There was a ribbon that I sewed on and then I thought “Oh, I like this thread. It's got sequins on it” and I thought “I'm going to sew that on” and then I thought “Wait a minute…How the heck am I going to sew this with the sequins on it?” But one of the facilitators had provided a very large needle so I persevered, and I was able to embroider “love” onto it. So, I was quite pleased that I was able to do that. It was neat to find the resources to do it. That's kind of a statement in itself, is not it? Something I was challenged with, but yet I was able to find a resource that enabled me to complete it. (Lynn, S2I).

Continuing with the theme of vulnerability and new perspectives, Donna described how showing her artwork to her granddaughter (see Figure 4) changed her perception. Based on her granddaughter's reaction, Donna decided that the artwork is about herself and for herself. Even after the workshop ended, the finished piece continued to inspire her as a place from which to grow:

When I showed [my artwork] to her, she said that she did not see the message, “You are the now” right away. I had to tell her about it because [the word] “now” is so far removed from the other words. And I thought about that a little bit, and I thought this has to be a piece for me, and maybe I have to think about and search for “now”. It's not easy. It's not simple. (Donna, S1I).

The article "Art-Based Workshops for Women: An Opportunity for Reflection on Identity and Transformation following Cancer Treatment" was published in 2023. Journal: Occup Ther Int.

### 4.3. Theme 3—Transforming: The Self

The women's self-reflections suggest they were involved in a transformative process. Reflecting on the words chosen in “You are the now”, Donna provided plausible reasons for her depiction of the words “no, no, no.” It appears her choice was not fully intentional and that she was still unravelling the meanings in her art after the workshops had ended. In this quotation, Donna appeared to take a stand. Through her cancer experience, she let go of her past self to embrace a more assertive identity:

That was probably from all the times since I've been diagnosed where I was told that I could not do something. Especially by my medical oncologist, but also by my husband. And it got to the point where I thought, I have to figure this out. I'm a senior citizen almost, and now I have to figure out what's important to me and not listen to the noes. And the noes may have some things in them that I have not thought about, but my medical oncologist did not want me to travel when I was first diagnosed and I was metastatic, and I said to my husband: “Now is the time to take our family on a family vacation. The future is now.” So, we booked a cruise in the Caribbean, and the oncologist argued with me for ten minutes about why I should not go, and I said: “I already booked a trip, and I'm going.” (Donna, S1I).

Patricia also described changes to the self as she discussed her deliberate use of symbols of the transformation she is going through, from a cancer patient to a healthy woman:

I did have an intention while making it, of that liberation and that cycle closing and transformation, inspiration. When you do art, you are always reflecting whatever's going on inside of you. (…) again, because of my cancer treatments being over, my intention was, “Okay … I'm turning into a butterfly now.” I'm not a sick person. I'm a healthy person and surrounding myself with light and… I do not have to be in that world of follow-ups and whatnot. Just become a normal person. For me, it was that idea of transformation that was there. Having seeds from plants, different seeds, it will become something else. Sort of a rebirth, new beginning, transformation. (Patricia, S2I).

The article "Art-Based Workshops for Women: An Opportunity for Reflection on Identity and Transformation following Cancer Treatment" was published in 2023. Journal: Occup Ther Int.

In short, the theme of transformation was described in various ways, but always in relation to the art-making process.

### 4.4. Theme 4—Creating: Regular Practices

Participants recognized the benefits of the workshops and often decided to incorporate elements of art-based occupations in their daily or regular practice. The finished artwork displayed in the homes of participants acted as reminders of the importance of taking care of oneself. “Karen” said the following:

The feeling that was created there, what I have been trying to do or craving is getting that feeling to come back. The mural above the bed (…) is a reminder to create that [feeling] again. I need to now create for myself that feeling [associated with the workshops] again in my life. That is what's happening every day, with everything that I'm doing. I'm trying to create that again, because that had such a positive effect on my wellbeing, mentally and physically. (Karen, S1I).

Similarly, in reflecting upon her experiences, Susan said the following:

What might've changed is that I'm taking a bit more time just to be. Not only in doing my artwork but also, I used to meditate regularly, and I started that again. [The workshops] reminded me that setting aside dedicated time to do something like meditation is a really good investment of my time and energy. (Susan, S1I).

Thus, for some participants, creativity was a part of a holistic approach to various, meaningful occupations. The intention to create on a regular basis may be read as indicative of the important role of creative practices and goals within occupational therapy.

## 5. Discussion

The aim of this study was to explore the experiences of women who are living with cancer and who participated in a series of mixed-media workshops while emphasizing themes of identity and transformation. Our analyses demonstrate that the workshops afforded participants' time to engage in pleasurable activities and provided opportunities to explore or revive an interest in creative practices. These findings support Maersk et al.'s assertion that art-based activities can bring joy and positive energy to women who experience cancer [21].

Over and above these outcomes, engagement in the art-based activities provided participants with an opportunity to reflect on their illness experience through states of flow and opportunities for self-expression and self-identification in the creative process. These findings support the literature asserting that art-based occupations have therapeutic potential for women to process their experiences with cancer. The women did not necessarily expect to draw such direct reflections of themselves from their art pieces. This is apparent in their surprise at the process of artmaking, the finished pieces, or what aspects of themselves they were able to see in them. In this sense, many participants were surprised by the depth of what was suggested through their artwork. This finding supports the claims that art-based occupations have the power to express familiar as well as more concealed feelings regarding self and the experience of illness [6, 12, 23, 28].

The article "Art-Based Workshops for Women: An Opportunity for Reflection on Identity and Transformation following Cancer Treatment" was published in 2023. Journal: Occup Ther Int.

Although such therapeutic experiences are thought to be essential to living well with cancer, opportunities to reconstruct the self are currently lacking in the care of women living with and beyond cancer [16, 18]. Taken with the processes used by facilitators to encourage self-reflection, these findings illustrate how art workshops have much to contribute to the practice of occupational therapy in the context of cancer survivorship. Indeed, occupational therapists are often found in group facilitating roles and have the necessary skills and knowledge to ensure a safe and accessible space to provide opportunities to engage in a therapeutic process through meaningful occupation [34].

### 5.1. The State of Flow and the Self

Our data demonstrate that the women were thoroughly engaged in the art-based activity which ultimately allowed for deeper reflections on the self. As noted above, this experience of complete engagement, for some, resembled the state of flow [24, 35]. From a period of flow, the self may emerge more prominently, providing the opportunity for further self-reflection and reconstruction [35]. The state of flow can be fostered by occupational therapists by providing a “just-right” challenge that invites confidence, control, and discovery [36]. Reynolds and Prior described the experiences of flow for women living with cancer participating in art-based occupations [11]. Similar to the experiences of our participants, the art-making process was described as enabling deep concentration, feelings of confidence, and the development of new skills related to a positive identity. After participating in the art-based workshops many women in our study stated their interest in incorporating art-based activities into their daily lives. Adding this new occupation to women's repertoire, or reminding them that such occupations are possible, could not only potentially address the occupational disruption caused by illness [16, 28] but also help build new and positive identities [11, 30]. Indeed, according to Dubouloz, engaging in immersive and reflective occupations can provide opportunities for clients to enter a process of change leading to positive transformation [19].

The article "Art-Based Workshops for Women: An Opportunity for Reflection on Identity and Transformation following Cancer Treatment" was published in 2023. Journal: Occup Ther Int.

### 5.2. Opportunities for Transformation

Perruzza and Kinsella [26], La Cour et al. [28], and Hansen et al. [25] all indicate that art-based occupations have an infinite potential for exploration and the consideration of new beginnings. Some participants indicated that their creations were stand-ins for themselves. Through reflection on their art pieces, they were able to understand in new ways their experience of cancer and see themselves in a new light. Drawing from Dubouloz Wilner's work on transformative learning theory in physical rehabilitation, it can be said that the art-based workshops provided the opportunity for critical self-reflection allowing for the examination of one's assumptions and the development or reconstructions of previously held meaning perspectives [13]. Donna's experience as described under the theme of *Transforming: The Self* demonstrates how a meaning perspective of valuing professional and familial advice was critically examined by the participant and reconstructed to embrace her own belief of having the ability to travel. A new meaning perspective of self-assurance and self-worth was then revealed. Although the change itself happened prior to the act of artmaking, the participant's reflection of her use of words such as “You are the now” and “No, no, no” displays a continuing process of self-reflection and the evolving process of meaning perspective development.

Dubouloz Wilner has urged rehabilitation professionals to make space for clients' “inner-voice,” thereby promoting self-reflection and transformation, given its centrality and importance in rehabilitation outcomes [13]. Occupational therapists are well-positioned to provide opportunities for occupations, such as art-based activities that allow for such a process to occur.

### 5.3. Focusing on the Activity Rather than the Words

Having a project to work on may have meant that it was easier for workshop participants to discuss with peers without having to directly address their illness. Our findings support the assertion that art-based activity groups direct the conversation to the creative process [23, 26, 29]. This emphasis might be welcome for those who are not interested in conventional cancer support groups.

Reynolds and Lim [27] as well as Perruzza and Kinsella [26] state that art-based occupations are suitable forms of self-expression when ideas are too challenging to put into words. In our study, the art-based activities presented in the workshops allowed study participants to freely explore their experience with cancer and their hopes for the future through creative materials. Using art as a means of self-expression removed the barrier of finding the words to communicate complex ideas that otherwise might not have been expressed or reflected upon.

The article "Art-Based Workshops for Women: An Opportunity for Reflection on Identity and Transformation following Cancer Treatment" was published in 2023. Journal: Occup Ther Int.

Facilitators invited but did not expect participants to share with the group what their art piece revealed about themselves or their cancer experience, although most did. Though they were disclosing personal information that could have made them feel vulnerable, this practice was perceived as nonthreatening since the women controlled what they shared. Haltiwanger et al. also assert that discussion-based peer groups are interpreted as more threatening than art-based groups [23].

### 5.4. Strengths and Limitations

Our research provides new indications as to the ways in which artists, occupational therapists, and others may collaborate to meaningfully support women living with the long-term effects of cancer. The project was not without limitations, however. While qualitative research is not meant to be representative, our sample was fairly homogeneous, particularly with respect to ethnicity. In addition, while the workshops were offered free of charge and were in an accessible, community-based location with free parking and easy access to a public transit hub, the workshops were offered on weekdays which could have precluded participation by those engaged with paid work or without childcare. Although no prior experience was necessary to participate in the workshops, it is possible that participants who enjoyed arts were drawn to the workshops and experienced greater benefits.

### 5.5. Implications for Occupational Therapy

Our study contributes to the occupational therapy literature by bringing to light the experiences of women living with cancer who have engaged in art-based occupations. We also help develop the still relatively small bodies of literature related to transformative occupations. This project blurred the lines between research and intervention. We utilized an occupational therapy lens to examine how a series of art-based workshops held for women living and aimed at enhancing their well-being could serve as an example of how engagement in meaningful occupations, such as art making, can provide clients with the opportunity for personal reflection and transformation. The positive experiences shared by the participants suggest the importance for occupational therapists to explore with their clients, meaningful occupations that can aid in the transformation of ideas regarding their personal illness experience. Many women living with cancer desire support not only during but also following traditional medical and rehabilitation phases, where they are faced with reconciling with new and disrupted identities. Occupational therapists may wish to use art-based activities to address the expression of identity and to process experiences related to cancer or chronic illness with women. This should be done in a safe and supportive environment with occupational therapists who have some experience with art-based occupations.

The article "Art-Based Workshops for Women: An Opportunity for Reflection on Identity and Transformation following Cancer Treatment" was published in 2023. Journal: Occup Ther Int.

## 6. Conclusions

Cancer has life-changing and enduring effects on the lives of women who experience it. Specifically, women living with cancer express that the need for support by healthcare professionals to help navigate the biographical disruption brought on by illness is lacking. Occupational therapists are well-positioned to provide such support through meaningful and transformative occupations. This study highlights the ways in which art-based workshops may offer a safe space for self-expression and reflection on changing identities for women who live with cancer, without necessarily having to resort to words. As Proust ponders, art distinguishes itself from other occupations because it has the power to release the expression of a true self. Engaging in art-based activities was not only seen as a pleasurable and therapeutic activity but also one that can provide opportunities to reconstruct parts of the self, leading to positive transformation. These transformative processes are integral to positive coping, management, and adaption to life-changing illness.

The findings point to ways occupational therapists can form new partnerships with other disciplines such as art therapists and the importance of our role in postrehabilitation settings to generate positive outcomes for people living with cancer. Future research could focus on the benefits of art-based occupations for cancer survivors and people living with chronic illnesses who have adopted a long-term creative practice or on the exploration of the characteristics of other occupations that offer means to deal with a life-threatening illness.

## Figures and Tables

**Figure 1:** A mixed-media project by a workshop participant.

**Figure 2:** Detail from a memory box.

**Figure 3:** Detail of the content from a bag after the turmeric bath.

**Figure 4:** “You Are the Now” detail from a mixed-media project by Donna.

**Table 1:** Participant summary.

Participants^1^	Age	Participation in workshop series	Cancer type and year of diagnosis
Ashley	43	1	Lymphoma and breast cancer (2013 & 2016)
Lynn	69	1 & 2	Breast cancer (2012)
Patricia	60	1 & 2	Breast cancer (2012)
Karen	60	1 & 2	Neuroendocrine cancer (2006)
Susan	72	1 & 2	Neuroendocrine cancer (2008)
Donna	(not disclosed)	1 & 2	Breast cancer (2010)
Sandra	57	2	Cervical cancer (2006)
Jessica	37	2	Breast cancer (2017)
Nicole	36	2	Brain tumour (2008 and 2016)
Erin	43	2	Breast cancer (2011)
Maya	35	2	Peritoneal mesothelioma (2014)

^1^Participants were assigned pseudonyms.

The article "Art-Based Workshops for Women: An Opportunity for Reflection on Identity and Transformation following Cancer Treatment" was published in 2023. Journal: Occup Ther Int.

**Table 2:** A detailed description of each workshop series.

	Workshop series 1	Workshop series 2
Structure	3 workshops (3 to 4 hours each)	3 workshops (3 to 4 hours each)
Description	The mixed-media workshops were facilitated by the PI and a professional visual artist at a local cancer centre. The facilitators emphasized the importance of embracing imperfection within the creative process. During the workshops, the facilitators played music and offered snacks and beverages during breaks. An abundance of material was provided and meant to inspire and guide the participants.	
Objective	Enhancing the well-being of women living with cancer via mixed-media art-based activities	
Theme	Wabi Sabi: “Finding beauty in imperfection”	Texturing small changes: “Small things can lead to big things”
Projects	Canvas painting Expressive collage on canvas Memory box Collage on textured boxes	Small canvas painting Seed canvas Turmeric bundle (participants used intuitive stitching on cotton bag holding photos, other images, and small mementoes; then, they were dyed in a turmeric bath) Copper brooch
Materials	Paint, pastels, watercolour pencils, ink, cardstock, lace, gauze, ribbons, threads and textured paper, pages from books and well-known sayings, illustrations, different fabrics, beads, feathers, shells, participants' own small meaningful objects…	Paint, pastels, watercolour pencils, ink, cardstock, lace, gauze, ribbons, threads and textured paper, pages from books and well-known sayings, illustrations, different fabrics, modelling paste, rusty metals, copper sheets, puzzle pieces, objects from nature (e.g., dried petals, twigs, pinecones, seeds, stones, and shells), participants' own small meaningful objects…
Guidelines	Each session began with an introductory exercise and presentation of the project suggested for the workshop. Examples of introductory exercises included the following: mark-making, haiku, journaling, thinking of song lyrics, meditation, visualization exercises, and reading selected quotations (e.g., from poetry). Following this, facilitators encouraged participants to work intuitively and freely, making suggestions rather than giving instructions. Throughout the workshops, the facilitators provided participants with artistic techniques and guidance as needed. Each workshop concluded with a group discussion during which each participant shared the work they had created.	
Number of participants	6	10

**Table 3:** Sample postworkshop telephone interview questions.

Interview questions
Do you find you are more or less able to make time for yourself as a result of this program? Was the art-making helpful in understanding your experience with cancer? In what ways? In coping with cancer? In what ways? Tell me about your creations. Do they represent your experiences with cancer? What are your thoughts about the group aspects of the program? Having talked about the workshop and cancer, can you tell me a bit about the impact of the workshop on your everyday life? For example, in terms of artmaking, self-care, and leisure?

The article "Art-Based Workshops for Women: An Opportunity for Reflection on Identity and Transformation following Cancer Treatment" was published in 2023. Journal: Occup Ther Int.

**Table 4:** Facilitation data.

Workshops	Facilitators' sample quotations
Workshop series 1	The main thing is to just relax and enjoy. It is a wonderful place to be, we are safe here with great people. And we are just really going to discover things. I just wanted to share this expression that I was thinking about. “Whether we are artists or scientists, craftsmen or tradesmen, philosophers or practitioners, we are all creators. We each create best when we use our total self, lending our body and our mind and our spirit” (professional artist). One of the things to do is to just take a moment, step back, and have a look at (the art piece) from another side of the room and then just giving it a little time, because the neatest thing is you can change it. Right, because I did that tree, and I decided no, I do not want that in there. So now you just listen to that voice inside that says, “What happens if I try this?” Or you might want to completely leave out an area, and that is perfectly all right, you are the creator (professional artist).
Workshop series 2	Because stories shift over time when you take them out next week, you might be like, “I do not remember…” this would be me, “I do not remember what I was thinking last week.” Or it might be, “well, that was an interesting story but since I've had time to think about it, I feel like this is telling me a different story.” So we are going to do something that involves a process of selection and story next week with all of these contents. So, this is not the end. Even if you have a very linear story and, as my co-facilitator said, it does not have to be, it will change next week with what's happened to the contents and what you pull out and how you are feeling and what you are thinking next week (principal investigator). This was an exercise that I did in a workshop called mending stories, it was a visual journaling workshop… the whole idea behind the workshop was that when you keep stories inside and you do not share them, then they have a lot of power to have negative effects on your lives. I am a researcher so there is probably some science behind that somewhere, but this was just the artist's beliefs so whether you want to buy into that or not, it is entirely up to you. But I do think that we have been storytelling as human beings for a very long time. So, there is power in story and getting stories out, you begin to mend the stories. So, there is a number of ways you can incorporate story into this bag. So, you all brought things in I see, and some people brought extra and that is wonderful (principal investigator).

The article "Art-Based Workshops for Women: An Opportunity for Reflection on Identity and Transformation following Cancer Treatment" was published in 2023. Journal: Occup Ther Int.

## Data Availability

Data are available from Roanne Thomas (roanne.thomas@uottawa.ca).
